The article "A Study on Credit Data-Based Poverty Alleviation in Rural Yunnan, China" was published in 2022. Journal: Comput Intell Neurosci.

# A Study on Credit Data-Based Poverty Alleviation in Rural Yunnan, China

**DOI:** 10.1155/2022/9498056

**Published:** 2022-08-22

**Authors:** Song Deng, Di Yang, Zhaoli Gao, Zhen Yuan, Chenghui Yao

**Affiliations:** School of Government, Yunnan University, Kunming, Yunnan 650091, China

## Abstract

The main path of development credit funds in rural poverty alleviation in Y province is crucial. This paper studies the rural poverty alleviation work in extreme poverty areas in Yunnan and puts forward targeted and instructive policy suggestions for specific difficult areas. Research the relationship between credit resource allocation and rural poverty alleviation. The existing research is mainly based on the relationship between financial development and economic growth, income growth, income distribution, and, on the surface, the relationship between the scale of financial development and the efficiency of financial development and other indicators. The purpose is to put forward targeted measures and suggestions on the basis of theoretical research and model analysis to help the Yunnan banking industry support poverty alleviation. The results of the study show that there is a causal relationship between agriculture-related loans.

## 1. Introduction

Poverty is a severe challenge facing China and has always received significant attention from the Chinese government. The “China Rural Poverty Alleviation and Development Program (2011–2020)” clearly put forward that by 2020, China should achieve the poverty alleviation of the rural poor and build a moderately prosperous society. Financial poverty alleviation plays an indispensable role in the current work, providing necessary support for poor areas to win the battle against poverty.

Foreign scholars have continued to focus on the correlation between financial development and poverty. While the classic ideas include the “vicious circle of poverty” and the “low-level equilibrium trap theory” proposed in the last century, international research on rural poverty alleviation has also made much progress in recent decades. Studies showed a positive relationship between rural financial development and poverty reduction [1, 2]. Esho argued that most of the financial poverty alleviation cooperatives in Australia are subsidized by the government and also pointed out that the size of the institution's deposit and loan is the main factor that determines the operating cost of the said financial poverty alleviation institutions [3, 4]. Geda et al. examined the relationship between finance and poverty using data on urban and rural households in Ethiopia from 1994 to 2000. The results show that people's use of financial products significantly smooths consumption and thus reduces poverty [5, 6]. Wang et al. pointed out that the main problem of difficulty in obtaining loans in developing countries is due to the inadequacy of formal financial supply and, on this basis, analyzed the main problems in the development of rural financial markets in underdeveloped countries [7]. Garedew et al. concluded that poor areas of financial service institutions face the main problem of cost when serving farmers. The core of solving the cost problem is to solve the inadequate information. At the same time, credit and social capital can provide support to solve the cost problem [8, 9]. Biswas and Saha analyzed the structure of rural commercial banks in the USA by constructing a dynamic model and pointed out that the US rural banking market is imperfectly competitive. The efficiency of bank operation is generally low [10–14]. They suggested that the rural commercial banks in the US farmers and that bank development policies promote competition in the rural financial market.

Xu and Gao studied the important influences on farmers' income increase and the correlation between these factors on supporting rural finance from the analysis of conceptual data on factors such as farmers' education level, farmers' credit investment, agricultural prices, and farmers' employment structure [15–17]. Cui and Sun used panel data from 1978 to 2010 to test the correlation between financial development and poverty alleviation. The results showed that financial development could increase the income level of the poor. However, financial fluctuations offset the poverty alleviation effect of financial development [18–24]. Huang pointed out in his article “Exploration on Anti-Poverty and Rural Financial System Arrangement” that the current rural financial system arrangement has problems, such as the impaired function of policy finance in anti-poverty, and proposed to build a rural financial system based on policy finance and cooperative finance as the main body [25].

This paper studies the rural poverty alleviation work in the extremely poor areas of Yunnan and puts forward targeted and instructive policy suggestions for specific difficult areas. Research the relationship between credit resource allocation and rural poverty alleviation. Existing research is mainly based on the relationship between financial development and economic growth, income growth, income distribution, and, on the surface, the scale of financial development and the efficiency of financial development and other indicators to study the relationship. The aim is to put forward targeted measures and suggestions based on theoretical research and model analysis to help the Yunnan banking industry support poverty alleviation.

## 2. Research Methods and Ideas

This paper proposes research hypotheses combining existing research results and practical experiences and verifies the relationship between credit resources in terms of scale (agriculture-related loan balance) and structure (industrial development category, fixed assets category, and technical services category) and the effectiveness of rural poverty alleviation through the model. The relationship between credit resource allocation and rural poverty alleviation effectiveness in the Yunnan banking supervision industry is supplemented with case studies to support further and corroborate the findings of the data model, taking into account the experience of banking supervision, daily research, and problems reflected by the operation process of banking institutions.

The specific research methods and ideas of the article study are shown in Figure 1.

## 3. Model Construction

### 3.1. Selection of Study Variables

The research variables in this paper involve both, that is, credit resource allocation and rural poverty alleviation effects.

In terms of the metrics of credit resource allocation, considering the actual situation of rural financial development in Yunnan Province and the integrity and reliability of financial statistics, we decided to select the relatively complete time series of year-end balance (AL) indicators of agriculture-related loans of all financial institutions in Yunnan Province. In order to further analyze the data and draw valuable research conclusions, this paper classifies the agriculture-related loan indicators in the original statistics into three categories according to the statistical caliber of the People's Bank of China and the nature of loan usage: first, loans for agriculture, forestry, animal husbandry, and fishery; agricultural materials and agricultural by-products circulation; and agricultural products processing are classified as industrial development loans (ALa); second, loans for rural infrastructure construction and farmland capital construction loans are classified as fixed assets loans (ALb); third, agricultural production materials manufacturing loans and agricultural science and technology loans are classified as technical service loans (ALc). The details can be seen in Table 1.

The specific contents of agricultural land capital construction loans include the following: agriculture, forestry, and fishery loans; agricultural materials and agricultural by-products circulation loans; agro-processing loans; rural infrastructure construction loans; farmland capital construction loans; agricultural production materials manufacturing loans; and agricultural science and technology loan.

In terms of the rural poverty alleviation effect metrics, the current national poverty line standard is RMB 2,300 (2010 constant price) per capita net income of farmers. Although the annual number of people removed from poverty directly reflects the effectiveness of poverty alleviation, there are specific problems in using the annual number of people removed from poverty as a metric to measure the effectiveness of rural poverty alleviation. On the one hand, the scientific nature of the indicator is lacking for academic studies. The number is more of an indicator preset at the beginning of the government's work report, which has the nature of a brutal government task; on the other hand, for the poor population, there is no substantial difference between the net per capita income of farmers of 2,400 yuan and 2,200 yuan for the living condition of the poor population.

This paper uses the original data of farm-related loans and farmers' net income per capita from 2010 to 2015. The rest of the data are obtained from the off-site supervision system of CBRC and the Kunming Central Branch of PBC and ensures the authority and high credibility of the data.

### 3.2. Formulation of the Research Hypothesis

As an essential component of rural finance, agriculture-related loans positively affect rural economic development and farmers' income growth. Although Cui and Sun studied the role of financial development on poverty alleviation using comprehensive national and provincial data [18], there is still logical uncertainty about whether the use of national data can fully explain the relationship between credit growth and net per capita income of farmers in Yunnan Province since this study is not entirely consistent with the variable system used in existing studies and the particular challenging provincial situation in Yunnan Province.

**Hypothesis 1 .**

(H1): There is Granger causality between farm-related loans and farmers' net income per capita.

Among the agriculture-related loans granted by banks, there are loans directly granted to farmers to engage in agricultural production activities such as agriculture, forestry, animal husbandry, and fishery; there are also loans similar to “to get rich, first build roads,” which do not work directly on farmers but on improving rural infrastructure construction such as transportation and drinking water or indirectly improving farmers' production and living conditions to alleviate poverty. There are also loans for technical services that aim to improve agricultural technology and equipment and farmers' technical skills. To ensure the rigor of the research results, this paper hypothesizes the effects of different types of farm-related loans on rural farmers' net income per capita.

**Hypothesis 2 .**

(H1a): Industrial development type loans have a significant positive effect on farmers' net income per capita.

The author takes industrial development loans as the primary indicator for analysis and research and aims to accurately reflect the actual effectiveness of credit resource allocation for rural poverty alleviation by the leading indicator of agriculture-related loans.

**Hypothesis 3 .**

(H1b): Fixed asset type loans have a significant positive effect on farmers' net income per capita.

The construction of infrastructure is of great importance in “poverty eradication.” In allocating bank credit resources, the primary credit investment includes the construction of critical infrastructures such as road transportation, water power grid, drinking water safety, and communication facilities in poor areas. The author recognizes the crucial role of fixed asset loans in rural poverty alleviation, so this paper singles out fixed asset loans as an essential part of credit resource allocation. The data include rural infrastructure construction loans and farmland capital construction loans in terms of fixed asset class loans.

**Hypothesis 4 .**

(H1c): Technical service type loans have a significant positive effect on farmers' net income per capita.

Technical services are an essential aspect of financial assistance to combat poverty. The traditional “blood transfusion” approach of giving money and goods alone will never work if farmers want to get out of poverty and become rich. Since 1986, the Chinese government has established a developmental approach to poverty alleviation. It has overhauled the traditional relief approach to poverty alleviation, shifting the national support strategy from the relief approach (“blood transfusion”) to the developmental approach (“blood creation”), placing more emphasis on education and education. The poor people use their hard-working hands and technical methods to embark on poverty alleviation and prosperity. This shows that singling out technical service loans as an essential aspect of credit resource allocation is necessary to reflect the effectiveness of rural poverty alleviation. The structure of technical service loans is shown in Table 2, including loans for manufacturing agricultural means of production and loans for agricultural science and technology.

### 3.3. Data Smoothness Test

According to the Statistical Bulletin of National Economic and Social Development of Yunnan Province, the per capita net income of farmers in Yunnan Province from 2010 to 2015 is shown in Table 3.

Due to the time constraints of the PBOC and CBRC in establishing the agriculture-related loan system, the data sample time series of this paper is for a total of six years from 2010 to 2015, as shown in Tables 4 and 5.

Since the data time series are not long, it is necessary to test the smoothness of the variables first before conducting the analysis. We used different ADF unit root tests according to the minimum criterion of AIC and SC taken in EVIEWS software to test the smoothness of AL, ANI, and their first-order differences AL1 and ANI1, respectively, and the results are shown in Table 6.

The test results show that the AL and ANI series are nonstationary, while their first-order differences are stationary. That is, they belong to the I(1) process. Similarly, the smoothness tests are performed for ALa, ALb, and ALc and their first-order differences, and the results are shown in Table 7.

The test data shows that the first-order differences of ALa, ALb, and ALc under AL for agriculture-related loans are all smooth and belong to the I(1) process to proceed to the next step of model analysis.

## 4. Empirical Analysis and Hypothesis Testing

### 4.1. Granger Causality Test

In this paper, the data were tested for smoothness. The results showed that the first-order linear combination of the data was smooth, reflecting the existence of a long-term stable proportional relationship between the variables (cointegration relationship). The tests performed on AL and ANI and their first-order differences are shown in Table 8.

From the Table 8, it can be seen that there is a correlation between the variables of credit resource allocation (represented by the balance of agriculture-related loans) and the variables of rural poverty alleviation (represented by the net per capita income of farmers) in Yunnan Province at the 5% and 10% significance levels, following which we further explore the specific causality situation.

According to the ECM model analysis method (the error correction model (ECM) was proposed by Davidson, Hendry, Srba, and Yeo in 1978.), the general expression of the ECM model for bivariate analysis is

(1) $$\begin{array}{c} d{\text{ANI}}_{1}=\alpha_{1}+\beta_{1}E+\sum_{t-l}^{t-1}\gamma_{i}^{1}d{\text{ANI}}_{1}+\sum_{t-k}^{t-1}\lambda_{i}^{1}d{\text{AL}}_{i}+v_{t},\\ d{\text{AL}}_{1}=\alpha_{2}+\beta_{2}E+\sum_{t-m}^{t-1}\gamma_{i}^{2}d{\text{ANI}}_{1}+\sum_{t-n}^{t-1}\lambda_{i}^{2}d{\text{ANI}}_{i}+\mu_{t}, \end{array}$$

where AL denotes the farm-related loan variable, ANI denotes the net income of rural residents variable, *d* denotes the first-order difference, and *E* is the residual value obtained by regressing the level quantities of these two variables with cointegrating relationships. Here, *E* is substituted into the model as the error correction term. The correlation results are obtained using the joint cubic system approach for trial calculations, as shown in Tables 9 and 10.

As shown in Tables 9 and 10, first, the error correction term is not significant in the credit resource allocation regression model, while the error correction term is significant in the rural poverty alleviation effectiveness regression model. This indicates that the long-run equilibrium relationship between the two results from Granger causality of the changes in rural poverty alleviation effectiveness caused by credit resource allocation in Yunnan Province. Second, in the rural poverty alleviation effectiveness regression model, none of its lagged terms are significant. Credit resource allocation is not significant except for 1 and 2, indicating that credit resource allocation in Yunnan Province has a time lag effect on rural poverty alleviation effectiveness, which is caused by the relatively long periodicity of agricultural production and the fact that the promotion effect of fixed asset and technical service loans does not appear immediately. This indicates that the short-term promotion effect of credit resource allocation for rural poverty alleviation is not significant and presents a long-term equilibrium relationship.

### 4.2. OLS Multiple Linear Regression Analysis

From the hypothesis of this paper, it can be seen that in addition to the scale of credit resource allocation on rural poverty alleviation in Yunnan, industrial development loans (ALa), fixed asset loans (ALb), and technical service loans (ALc) in the credit resource allocation structure also have a positive effect on the effectiveness of rural poverty alleviation, but how much each of these three indicators contributes to the improvement of rural poverty needs further research. Therefore, referring to Xu and Gao [15], this paper constructs a double logit model design as follows:

(2) $$\begin{array}{c} y=\text{KAL}a^{\alpha }\text{AL}b^{\beta }\text{AL}c^{\nu }, \end{array}$$

where *y* is the per capita net income of rural residents, an indicator of rural poverty alleviation effectiveness; *K* is a constant item *K* > 0; ALa is the loan balance of the industrial development category; ALb is the loan balance of fixed assets category; ALc is the loan balance of technical services category; and *α*; *β*; *ν* are parameters. It can be seen that an increase in any one of these factors will lead to an increase in the net income of rural residents, with other conditions held constant, and this model is consistent with the assumed premises of the text.

If we take the logarithm of both ends of (2), we get

(3) $$\begin{array}{c} \text{IN}y=InK+\alpha In\text{AL}a+\beta In\text{AL}b+\nu In\text{AL}c. \end{array}$$

The above model is thus transformed into a multiple linear regression model style, and we can use the OLS method (OLS is short for ordinary least square. Ordinary least squares estimation is to find the estimates of parameters *β*1, *β*2… such that the sum of squares of the departures from the above equation *Q* is extremely small. Each squared term in the equation has the same weight and is an ordinary least squares regression parameter estimation method. Under the condition that the error terms are equal variance and uncorrelated, ordinary least squares estimation is a linear unbiased estimate of the minimum variance of the regression parameters) for regression analysis. Here, *α* is the credit resource allocation elasticity of industrial development loan balances, and similarly, *β*; *ν* are the credit resource allocation elasticity of fixed asset loan balances and technology service loans, respectively.

(4) $$\begin{array}{c} \text{Denote }y1Iny;\;A1=In\text{AL}a;\;B1=In\text{AL}b;\;C1=In\text{AL}c;\;K1=InK. \end{array}$$

First, the single factor of rural industrial development type of loans and rural residents' net income were selected for regression analysis using the OLS method, and the results were as follows (the *t*-values of the coefficients are in small brackets):

(5) $$\begin{array}{c} y1=6.652+0.872A1\left(32.764\right)\left(14.125\right),\\ R2=0.935\;\bar{R^{2}}=0.921\;F=143.51,\\ y1=2.896+0.725B1,\left(12.003\right)\left(11.361\right),\\ R2=0.894\;\bar{R^{2}}=0.878\;F=98.32,\\ y1=2.896+0.625C1\left(12.003\right)\left(9.169\right),\\ R2=0.813\;\bar{R^{2}}=0.837\;F=67.17. \end{array}$$

From the above regression equation, it can be seen that the growth of net income per rural resident since 2010 has a strong correlation with the loan input in the rural industrial development category, with the largest correlation coefficient and the highest goodness of fit of its equation (*R*^2^ = 0.935). The elasticity of rural residents' per capita net income on the allocation of credit resources for industrial development is also relatively large, that is, each point of credit resources invested can bring about a 0.872 percentage point increase in rural residents' per capita net income. And the *t*-value of the coefficient is 14.125, which is much larger than the test value of *t*0.995 = 4.946, indicating the existence of linear correlation.

## 5. Policy Suggestions for Yunnan Banking Industry to Optimize Credit Allocation to Help Poverty Alleviation

Based on the findings of this paper's empirical test and combined with the current problems of poverty alleviation in Yunnan Province, the following suggestions can be made to improve the quality and efficiency of poverty alleviation credit allocation in Yunnan's banking sector.

### 5.1. Accelerate Industry Cultivation and Development

According to the study's conclusion, the key to poverty alleviation and development should rely on industry, through industrial development to drive farmers to increase income and enhance the “blood-making” function of poor areas themselves. First of all, government departments in poor areas should closely focus on the overall plan of eight key industries development in Yunnan Province based on local resource advantages; closely follow the market demand; develop highland agriculture, resource processing, rural tourism, and other special industries according to local conditions; turn resource advantages into economic advantages; and accelerate the accumulation of capital and the pace of poverty alleviation and wealth. Second, banking financial institutions should take the initiative to dovetail with poverty alleviation industrial projects, study and formulate financial service planning and specific measures to support the development of poverty alleviation industries, help cultivate several agricultural industrialization “small giants” and agricultural professional cooperatives, and help introduce leading agricultural enterprises and agricultural by-product acquisition enterprises. On the premise of risk control, actively innovate financial products; increase the investment of loans, microenterprise cultivation loans, and guaranteed business loans; and give microcredit support to poor families for opening online stores. Again, for industrial development poverty alleviation projects, according to the actual situation of enterprises, enhance the credit method based on the industrial poverty alleviation chain. Finally, to establish and improve the various types of poverty alleviation project fund matching platforms, improve the supporting financial services for modern agricultural industrial parks, characteristic advantageous industrial bases, and so on and increase credit support for new agricultural business entities such as farmers' professional cooperatives in poor areas to drive poor farmers to increase production and income.

### 5.2. Efforts to Break the Bottleneck of Infrastructure Constraints

Most poor areas lag in infrastructure and basic public service construction, which has become a great shortcoming in the fight against poverty. Governments at all levels should increase investment in key infrastructure projects in poor areas, give funds and projects in favor of enhancing the ability of poor areas to develop themselves and open up the “last mile” to get rid of poverty and get rich. First, we should actively play a complementary role in policy finance and commercial finance, and strongly support the construction of transportation facilities, information networks, energy security, safe drinking water, health care, and other projects in poor areas to promote access to water, roads, electricity, and communications and improve the living conditions of the poor. Second, we should focus on protecting the financial needs of water conservancy construction, improving production and living conditions in poor areas, and enhancing the support capacity of regional development. Third, we should strongly support the relocation projects for poverty alleviation, make good use of special construction funds, and increase credit support to implement all stages of poverty alleviation. Fourth, we should increase credit support for key projects in poor areas; actively follow up on agricultural surface pollution, soil pollution prevention and control, and agricultural waste harmless treatment projects; and promote ecological protection and restoration in poor areas.

### 5.3. Moderate Increase in Investment in Science and Technology Services

It is better to teach people to fish than to give him a fish. Increase the investment in “helping the wisdom,” help the poor people to master the skills to get out of poverty, increase the means of science and technology to get out of poverty, and be conducive to promoting long-term, sustainable poverty alleviation. On the one hand, governments at all levels should actively promote science and technology and intellectual poverty alleviation; combine science and technology with other production factors; fully mobilize the enthusiasm and creativity of the majority of scientific and technological personnel; vigorously develop rural vocational education, increase scientific and technological training; train farmers to master advanced practical technology; improve the use rate of resources and scientific and technological productivity, especially to actively increase the investment in education and poverty alleviation credit; improve the policy of student origin student loans policy; issue student loans to poor households with students studying in colleges and universities; subsidize the interest during the study period by the finance; and extend the loan period appropriately.

On the other hand, banking financial institutions should increase investment in financial resources for technical services and strongly support the transformation and upgrading of production materials, agricultural science and technology development, construction of science and technology demonstration parks, and vocational skills training in poor areas.

### 5.4. Sound Risk Compensation Mechanism

According to the study's conclusion, the investment in poverty alleviation loans has a significant positive impact on farmers' per capita net income. However, in practice, as the target of poverty alleviation loans are mainly low-income poor farmers, their repayment ability and risk resistance are weak, and the credit risk is large, which is not in line with the bank's sound business goal of “risk control and commercial sustainability.” According to the survey, only 93 poor counties (including provincial poor counties) in Yunnan Province have established a risk compensation fund for poverty alleviation.

Most counties have only 5 million risk compensation funds, which is measured by the 5 times magnification bar multiplier stipulated in the relevant policies. The risk compensation fund is mismatched with the demand for poverty alleviation loans. In addition, the risk compensation fund also has problems such as untimely disbursement of government subsidy funds, and the subsidy period is shorter than the production cycle of the breeding industry. Therefore, the government should improve the risk compensation mechanism for poverty alleviation loans as soon as possible, promote the compensation fund to cover all counties with poor populations, timely replenish the risk compensation gap, and amplify the leverage of financial funds and the function of poverty alleviation. The development and reform, poverty alleviation, finance, and other departments in poor counties should regularly inform the planning information of the region's characteristic industrial development, infrastructure and basic public services to the People's Bank of China, banking supervision, and all relevant banking institutions so that banking institutions can accurately grasp the project arrangements, investment scale, funding sources, schedule, and other information and accurately support the poverty eradication efforts according to the list of financial service needs.

### 5.5. Improve the Information Sharing Platform

During the research of this paper, the author found that it is very difficult to obtain specific data such as the number of poverty alleviation population and income changes of the poor in Yunnan Province, which reflects the side that there is a problem of information asymmetry between poverty alleviation departments and financial departments, which not only leads to the inefficiency of information transmission and use but also may cause banking institutions to face poor policy connection and incomplete information to carry out financial poverty alleviation work, which in turn leads to financial precise poverty alleviation. Therefore, it is necessary to further improve the information exchange and working linkage mechanism among the government, poverty alleviation, finance, human bank, banking supervision, development and reform, banks, and so on, to strengthen policy interaction, working linkage, information sharing, and coordination, to facilitate banking institutions to accurately match the financial service needs of various fields and effectively enhance the implementation effect of financial policies for poverty alleviation.

## 6. Concluding Remarks

### 6.1. Key Findings

Based on literature research and data collection, this paper conducts a study on rural poverty alleviation in Yunnan Province based on credit data from the banking sector in Yunnan Province. By comparing the relationship between rural-related loans and industrial development category, fixed asset category, and technical service category loans under rural-related loans and rural residents' net per capita income from 2010 to 2015, and constructing a model for Granger causality test and OLS multiple linear regression analysis, the following conclusions are drawn.

1. There is a Granger causality relationship between agriculture-related loans and farmers' per capita net income; industrial development loans have a significant positive impact on farmers' per capita net income; fixed asset loans have a significant positive impact on farmers' per capita net income; and technical service loans have a significant positive impact on farmers' per capita net income
2. At present, among industrial development, fixed asset, and technical service loans under agriculture-related loans, the most significant impact on farmers' per capita net income is on industrial development loans, followed by fixed asset loans, and the relatively insignificant impact is on technical service loans
3. In terms of public policy, it needs to be improved in terms of accelerating industrial cultivation and development, breaking the bottleneck of infrastructure constraints, increasing investment in science and technology services, improving information sharing platforms, and sound risk compensation mechanisms

### 6.2. Research Outlook

The positive effect of bank credit on improving the per capita net income of rural residents is demonstrated from two aspects of credit scale and credit structure, but this paper has certain limitations. First, the continuity of poverty alleviation data related to the banking industry is limited, and the statistical coverage needs to be further improved. Some statistical indicators have not yet been included in the scope of data collection. This paper fails to obtain time series data for a long period of time, nor to obtain specific data such as changes in the income of the poor, resulting in a lack of data stability in the empirical analysis; second, due to space limitations, this paper does not further demonstrate the impact of credit support efficiency on rural areas in Yunnan Province. The effect of poverty alleviation has not been studied on the optimal path for the allocation of credit resources in the province. There is no research on the optimal path of credit resource allocation in the whole province, which can be used as a further research direction for follow-up research.

## Figures and Tables

**Figure 1:** Research methods and ideas of this paper.

**Table 1:** Agricultural-related credit resource allocation index system.

Tier 1 indicators	Secondary indicators	Specific indicators for agriculture-related loans
Agricultural-related loans	Industrial development loans	Agriculture, forestry, and fishery loans
		Agricultural materials and agricultural by-products circulation loans
		Agro-processing loans
	Fixed asset class loans	Rural infrastructure construction loans
		Farmland capital construction loans
	Technical service loans	Agricultural production materials manufacturing loans
		Agricultural science and technology loan

**Table 2:** Summary of research hypotheses in this paper.

Assumption no.	Explanatory variables (credit resource allocation)	Explained variable (rural poverty alleviation effectiveness)
H1	Agricultural-related loans (AL)	Granger causality
H1a	Industrial development type loans (ALa)	Significant positive relationship
H1b	Fixed-asset-based loans (ALb)	Significant positive relationship
H1c	Technical service loans (ALc)	Significant positive relationship

**Table 3:** Per capita net income of farmers in Yunnan Province, 2010–2015.

Year	2010	2011	2012	2013	2014	2015
Revenue (yuan)	3,952	4,722	5,417	6,141	7,456	8,242

**Table 4:** Agricultural-related loan data, 2010–2015.

Loan purpose	Loan balance (billion yuan)					
	2010	2011	2012	2013	2014	2015
Agriculture, forestry, and fishery loans	905.92	685.39	777.72	855.65	967.56	1,039.17
Agricultural materials and agricultural by-products circulation loans	221.82	227.91	280.85	336.91	401.50	440.92
Rural infrastructure construction loans	956.36	1,096.37	1,159.84	1,062.73	1,160.43	1,190.29
Agro-processing loans	118.58	146.36	160.05	172.17	211.67	240.76
Agricultural production materials manufacturing loans	184.58	187.10	234.18	181.77	197.74	189.25
Farmland capital construction loans	125.90	141.07	116.83	118.15	95.92	134.55
Agricultural science and technology loan	14.63	11.60	16.84	11.60	8.24	5.03
Total farm-related loans (excluding others)	2527.78	2,495.79	2,746.30	2,738.98	3,043.07	3,239.97

**Table 5:** Agricultural-related loan data after categorization by loan nature.

Loan classification	Loan balance (billion yuan)					
	2010	2011	2012	2013	2014	2015
Industrial development loans	1,246.32	1,059.66	1,218.62	1,364.73	1,580.73	1,720.85
Fixed asset class loans	1,082.25	1,237.43	1,276.66	1,180.88	1,256.35	1,324.85
Technical service loans	199.21	198.70	251.02	193.37	205.98	194.28
Total farm-related loans (excluding others)	2,527.78	2,495.79	2,746.30	2,738.98	3,043.07	3,239.97

**Table 6:** AL and ANI variables smoothness test.

Variables	ADF test value	Inspection type	1% Critical value	5% Critical value	10% Threshold	Conclusion
AL	−2.223592	(C, 0, 1)	−4.887	−3.8377	−3.3677	Nonstationary
AL1	−3.424131	(0, 0, 1)	−2.6491	−1.9745	−1.6503	Flat at 1% level
ANI	0.164814	(0, t, 3)	−2.8376	−1.9653	−1.6241	Nonstationary
ANI1	−2.053887	(C, 0, 1)	−2.7986	−1.9654	−1.6301	Steady at 5% level

**Table 7:** Tests for smoothness of ALa, ALb, and ALc variables.

Variables	ADF test value	Inspection type	1% Critical value	5% Critical value	10% Threshold	Conclusion
ALa	−2.223592	(C, 0, 3)	−3.5203	−2.9878	−2.8797	Nonstationary
ALa1	−1.867342	(0, 0, 1)	−2.4332	−1.5643	−1.4689	Flat at 1% level
ALb	0.156832	(0, 0, 2)	−2.6735	−2.3561	−2.8751	Nonstationary
ALb1	−1.560932	(C, 0, 1)	−2.6591	−1.9782	−1.66431	Steady at 5% level
ALc	−3.856342	(0, 0, 2)	−3.2117	−2.5649	−2.4198	Nonstationary
ALc1	−2.017843	(0, t, 1)	−2.7531	−1.8796	−1.5493	Flat at 1% level

**Table 8:** AL1 and ANI1 cointegration test.

Variable	ADF test value	Inspection type	1% Critical value	5% Critical value	10% Threshold
Residuals *e*	−1.978712	(0, 0, 1)	−2.766	−1.9543	−1.5761

**Table 9:** Results of the Granger causality test for ANI1.

Explained variables	ANI1	
Variables and constant terms	Parameter estimates	*t*-test value
Constant term	−0.0557372	−1.376523
Error correction term *e*	0.969778	4.436712
AL1 (–1)	3.214532	3.097415
AL1 (–2)	1.537621	2.598719
Goodness-of-fit value	0.7951623	
Durbin–Watson test value	1.7035621	

**Table 10:** Results of the Granger causality test for AL1.

Explained variables	AL1	
Variables and constant terms	Parameter estimates	*t*-test value
Constant term	0.0318752	0.597651
Error correction term *e*	−0.056201	−0.1508319
ANI1 (–1)	0.286514	2.915632
AL1 (–1)	0.497153	2.801653
Goodness-of-fit value	0.685132	
Durbin–Watson test value	1.726531	

## Data Availability

The figures and tables used to support the findings of this study are included in the article.
